# Construction and Analysis of a Novel Wearable Assistive Device for a Visually Impaired Person

**DOI:** 10.1155/2020/6153128

**Published:** 2020-10-15

**Authors:** Shahid Akram, Ali Mahmood, Ihsan Ullah, Muhammad Tahir Mujtabah, Ali Bin Yasin, Asif Raza Butt, Muhammad Shafique, Sajjad Manzoor

**Affiliations:** ^1^Department of Electrical Engineering, Mirpur University of Science and Technology (MUST), Mirpur, 10250 AJK, Pakistan; ^2^Department of Electrical Engineering CUI, Abbottabad Campus, Abbottabad, KPK, Pakistan; ^3^Department of Biomedical Engineering, Riphah International University, Islamabad, Pakistan

## Abstract

In this paper, we have given the design and development of a new wearable device that assists visually impaired individuals to travel independently and confidently. The newly proposed device is based on range-based sensors and would work effectively in both indoor and outdoor conditions. It is constructed in the form of two separate modules; one module is designed such that it can be attached to the waist belt of the user, and the other module is designed to wear it on ankle of the user. Both the modules communicate with each other using wireless communication and can cover the full front environment of the user. The information about the front environment is transmitted to the user, via headphone, by sending a set of voice instructions, stored in a memory card added in the belt module. In order to use the device in crowd mode, appropriate networking techniques were also implemented in the prototype such that the interference of two or more devices in the close vicinity can be avoided. In the end, effectiveness of the device is analyzed and proved by conducting experiments and obtaining statistical results.

## 1. Introduction

With the advances in technology, commercial hardware and software applications are developed to make life easy for people with physical weakness. At least 2.2 billion people of the world have a vision impairment or blindness [1]. They may belong to a category, with moderately visually impairment, severely visually impairment, or totally blind. Most of the visually impaired people move by using conventional methods, i.e., white canes, guide dogs, tactile paving, and in some other cases move with the help of another person, called as sight guide [2, 3]. With the evolution of technology, there is an immense need for the development of easy-to-use devices that would be helpful for the visually blind people in mobility. In this way, visually impaired individuals may travel independently with confidence and participate in daily activities.

Recently, many types of electronics travel aids (ETA) have been developed for mobility assistance of blind people [4–6]. In Figure 1, different assistive devices for the blind are shown, which can be helpful during the motion of the user. The ETAs use sensors to detect obstacles in front of their users and give information about the front environment and guide the user in a manner that they would safely move forward. In some other devices, cameras are used for vision-based assistance of their user during motion. In some cases, Raspberry Pi cameras [7] are used to detect objects in front, and in other cases, Kinect sensors [8] are used to calculate the distance of the user from the obstacles. Smartphone camera-based elevator finder application was developed in [9]. This would help users to find if they are moving in the direction of the elevator or not. Mobile phone camera, with color codes was used in [10] in order to convey information about the inside of a building. In [11], the authors have used fusion of artificial vision and GPS for locomotion assistance and obstacle detection for the user. Fusion of ultrasonic sensor, GPS, and GSM was introduced in a silicon glove in [12]. A walking stick that uses radiofrequency identification (RFI) was constructed in [13] in order to help blind people navigate on their sidewalk. However, most of the assistive device for blind uses range-based sensors, which are cost effective, have good availability, and easy to operate. These user friendly devices use IR sensors [14], for small range; ultrasonic sensors [15, 16], for medium range; and/or LIDAR [17], for long range, to detect and localize obstacles in front of the user.

Most of the assistive devices for the blind, developed, till now, are either very costly or bulky for the user to wear or hold. The conventional white cane is already heavy and addition of any device on it can make it more difficult to hold. Vision-based devices, with cameras attached to them, mostly belong to the categories that are both heavy and expensive. These days, small cameras are available; however, cost remains the matter of concern in them. Similarly, smartphones, which are used in some applications for assistance for visually impaired, are also expensive. The devices based on ultrasonic sensor or any other range-based sensors do not cover all the features of the front environment. In order to solve all the issues, mentioned above, in this paper, we have proposed an assistive device for the blind which is inexpensive and lighter in weight. It is a wearable modular device. It is equipped with range-based sensors. These modules can be attached to the waist belt and the ankle of the user. This device covers more area in front of the user and is effectively helpful for his mobility. The experimental analysis on the device is also done to check its effectiveness.

This paper is further organized as follows: in Section 2, the purpose for the design and development, along with considerations taken during design phase of the new device for visually impaired person, are given. The architecture as well as the components used in the device is also discussed in this section. The algorithm designed for working of the device is given in Section 3. The model for the state estimator is discussed in Section 3.1. In Section 3.2, we have considered the issue of communication within the device in the crowd mode, i.e., crowded environment with multiple users at same place. In Section 4, the experimental and statistical results of the device are given, so that the effectiveness of the device for visually impaired people can be evaluated. Finally, in Section 5, the conclusion of the paper is given. The expected future development in the proposed device is also discussed in this section.

## 2. An Assistive Device for Visually Impaired People (aVIP)

Design, construction, and development of a new assistive device for visually impaired people are given in this section. One of the intentions of the research is to develop a cost-effective assistive device for visually impaired people.

### 2.1. Design Consideration for Assistive Device

During the design phase of the device, the following considerations were made to get maximum information about the front environment:

(1) The device should determine all obstacles in front of the user body, from the ground to the head, as shown in Figure 2(a). It should be able to distinguish obstacles at the following locations:
  - Large obstacles in front of the user, as shown in Figure 2(b)
  - Holes and pits, on the ground, in front of the user, as shown in Figure 2(c)
  - Hanging or inclined obstacles at the level of the head of the user, as shown in Figure 2(d)
  - Small object or stairs in front of the user, as shown in Figure 2(e)
  - Hollow objects (i.e., tables and chairs) in front of the user
(2) Information about the environment, in front, should be given in the form of a clear voice instructions.
(3) The instructions should be easy to understand; this could be recorded in the user's own voice.

In Figure 2(a), the layout of the proposed device is given that would accomplish all of the abovementioned tasks. A modular device, consisting of two modules with four different proximity sensors, is proposed. More detail of the architecture of the proposed device is discussed in Section 2.2.

### 2.2. Architecture of aVIP Device

In order to cover the maximum area in front of the user, the device is designed in a modular form by combining sensors, commercially available microprocessors, transmitter, and receiver. The architecture of the device is given in Figure 3. It is subdivided into two modules that communicate with each other without any wire. These modules are named as

- Belt module
- Ankle module

The belt module (BM) is designed in such a way that it can be attached to the waist belt of the user. The architecture of the belt module is shown in Figure 3. It serves as the master module for the ankle module (AM), and it has its own rechargeable power supply. This module has three ultrasonic sensors targeted in different directions. The first sensor is directed normal to the user body, and it would detect any obstacles in front of the user. The second sensor is directed in upward direction at an angle of 45° from first sensor. This sensor can detect obstacles only at head level such as lower roof or lower inclined side of the stairs. A third sensor is adjusted in such a way that it is directed downward at an angle of -45° from the first sensor. It can detect any pits or hole in the ground in front of the user. It would also detect any obstacle of small size or step, not detected by the first sensor. However, due to its orientation, the sensor would only be able to detect small obstacles such as step or footpath unless the user reaches very close to it. In combination with the ankle module this sensor would also detect small, hollow obstacles, i.e., tables and chairs. The developed belt module is given in Figure 4(a).

The belt module has two, commercially available, Arduino Mini microprocessors, connected with each other. This is due to the reason that each Arduino Mini has only one SPI interface while the belt module needs two SPI interfaces, i.e., one for a SD card that stores audio instructions and other for a communication device. The memory card is connected to one of the microprocessors. This memory card would have audio instructions recorded in it, each as a separate audio file. A headphone is also connected to the device through an audio amplifier. An nRf24L01 module acting as a receiver is connected to the other microprocessor in the belt module, so that the information from the ankle module can be wirelessly received.

The architecture of the ankle module is also shown in Figure 3. It has a single Arduino Mini microprocessor connected to a rechargeable battery. It has one ultrasonic sensor in it which is directed in the direction perpendicular to the user body. This sensor can detect all the obstacles of small size, which are undetectable to the sensors in the belt module. An inertial measurement unit (IMU) sensor is attached to the module to detect the dynamics of leg motion and differentiate straight and bent leg during swing or stance phase of motion. Using the IMU sensor, only obstacles in front of the user would be detected and the ground would not be considered as an obstacle when the leg would be in bent position. It can also be used to count the number of steps taken by user. The data from the ankle module is transmitted to the belt module through the nRF24L01 module. The nRF24L01 module in the belt module acts as a receiver while the one in the ankle module acts as a transmitter. The constructed ankle module is given in Figure 4(b)).

## 3. Working of the Device and Algorithm for Obstacle Detection

There are three ultrasonic sensors installed at waist height to measure the distance to the ground or an obstacle. One is installed normal to the body of user, the other up waist at 45°, and the third down waist at an angle of negative 45°-down to normal. The device installed on the ankle has an ultrasonic sensor directed normal to the body as well as an IMU. The belt and ankle modules detect the obstacle separately. However, only the belt module has an SD card connected to it that contains audio instructions for the user about the nature of the obstacles in front. Furthermore, headphones are also connected to belt module. Therefore, the belt module acts as the master and the ankle module acts as a slave.

All the sensors perform differently under different terrains and scenarios. Some of the common scenarios that a subject may face have been evaluated and considered in the design of the hardware, as shown in Figures 2(b)–2(e). The outputs from all the sensors are used to warn the user about any obstacle ahead. The first sensor to register this kind of obstacle will be the normal sensor. In case of a hole on a leveled surface, the primary action or warning is given to the user based on the input from the waist down sensor; however, the ankle sensor with IMU sensor output can be used to navigate the obstacle and scan the obstacle for clearance. In the scenario of the leveled surface with obstacle at head level only, up waist sensors gives distance. While in the case of stairs or small obstacle ahead, the normal sensor is again the first sensor to register an obstacle, but the classification of the obstacle can only be performed by the down waist sensor and the ankle sensor.

The outputs of sensors are passed through a moving average filter before using them for a decision. Since the moving average filter is also a low-pass filter, it smoothens any abrupt transitions thus eliminating any noise or erroneous measurements. The moving average filter implemented in the hardware is depicted in Figure 5. The assistive device has two modes of operation: setting mode and working mode. Same obstacle detection distance limits *l*_*b*_(limit) and *l*_*a*_(limit), for the front sensor in the belt and ankle modules, respectively, can be adjusted for the users of different heights. Therefore, there is no need to change these parameters. However, obstacle detection distance limits *l*_*h*_(limit) and *l*_*g*_(limit) for the respective head and ground sensors in the belt module can be affected by the height of each user. Therefore, whenever a user wears a device for the first time, it should be operated in setting mode to adjust these limits. During the setting mode, the user is instructed to stand on a plane surface and hold a plane paper sheet at head level. By pressing setting switch, the device would automatically adjust obstacle detection distance limits *l*_*h*_(limit) and *l*_*g*_(limit) for the head and ground levels. In order to avoid false detection due to uneven ground, small clearances *ϵ*_1_, *ϵ*_2_, and *ϵ*_3_ are added in the algorithm. Once the setting is done, the setting mode is closed and the device is operated on working mode. For instantaneous values *l*_*b*_, *l*_*h*_, and *l*_*g*_ of the respected normal, head level, ground level sensors in the belt module and values *l*_*a*_ of ankle sensor, the algorithm for operation of the assistive device is given in Algorithm 1.

### 3.1. The State Estimation Process

Since the measurements, especially for moving obstacles, are of stochastic nature, a Kalman Filter (KF) can be deployed for target state estimation. The measurement from the sensor consists of range *R*, to the moving object, i.e., *z*_*k*_ = *R* the time to react, *τ*, is not estimated for a few initial scans; afterwards, it is initialized from the estimated range and range rate and is made part of the filtering process. The final state propagates in discrete domain by

(1) $$\begin{array}{c} \chi_{k}=\phi \chi_{k-1}+U_{k}+w_{k}, \end{array}$$

where *χ*_*k*_ is the state vector, *U*_*k*_ = [0 0 *T*]^*T*^ and the plant noise, *w*_*k*_, is assumed to be white Gaussian noise with zero mean. The plant noise is characterized by a known covariance matrix *Q*. The state vector consisting of the range, *R*, range rate $\dot{R}$, and time to react, *τ*, is defined as

(2) $$\begin{array}{c} \chi ={\left[\begin{array}{ccc} R & \dot{R} & \tau \end{array}\right]}^{T}. \end{array}$$

The state transition matrix *ϕ* in Equation (1) is given as

(3) $$\begin{array}{c} \phi =\left[\begin{array}{ccc} 1 & T & 0\\ 0 & 1 & 0\\ 0 & 0 & 1 \end{array}\right], \end{array}$$

with *T* being the sampling time. The plant noise covariance matrix *Q* can be expressed as

(4) $$\begin{array}{c} Q=q.\left[\begin{array}{ccc} \frac{T^{4}}{4} & \frac{T^{2}}{2} & 0\\ \frac{T^{2}}{2} & T^{2} & 0\\ 0 & 0 & \frac{T^{8}}{8} \end{array}\right], \end{array}$$

where process noise variance is denoted by *q*. The KF update and prediction equations as given in literature [19] can be expressed as

(5) $$\begin{array}{c} {\hat{\chi }}_{k/k-1}=\phi {\hat{\chi }}_{\left(k-1\right)/\left(k-1\right)}+U_{k}+w_{k}. \end{array}$$

With

(6) $$\begin{array}{c} {\hat{\Gamma }}_{k/k-1}=\phi {\hat{\Gamma }}_{\left(k-1\right)/\left(k-1\right)}\phi^{T}+Q, \end{array}$$

the estimation part can be written as follows, where first we compute the innovation covariance matrix by

(7) $$\begin{array}{c} \xi_{k}=H_{k}^{\chi }{\hat{\Gamma }}_{k/\left(k-1\right)}H_{k}^{\chi^{T}}+R, \end{array}$$

where *R* is the measurement variance and is computed from the three-sigma bound of the sensor. The Kalman gain is given by

(8) $$\begin{array}{c} \Delta_{k}={\hat{\Gamma }}_{k/\left(k-1\right)}H_{k}^{\chi^{T}}+\xi_{k}^{-1}, \end{array}$$

such that, the estimated state vector can now be calculated from the Kalman gain and the measurement residue as

(9) $$\begin{array}{c} {\hat{\chi }}_{k/k}={\hat{\chi }}_{k/\left(k-1\right)}+\Delta_{k}\left(z_{k}-H_{k}^{\chi }{\hat{\chi }}_{k/\left(k-1\right)}\right). \end{array}$$

Finally, the state covariance matrix is computed by the following equation:

(10) $$\begin{array}{c} \Gamma_{k/k}=\left(I-\Delta_{k}H_{k}^{\chi }\right)\Gamma_{k/\left(k-1\right)}. \end{array}$$

The plant covariance matrix is initialized based on the process explained in [20]. The quality of the estimate depends on the sampling time *T* along with the assumed measurement process noise covariance matrix *R* and process noise variance *q*.

### 3.2. Crowd Mode Communication

The nRF24L01 chip is used for communication purpose, between two modules of the constructed assistive device [21]. It is a radio transceiver with a frequency operating range of 2.4-2.5 GHz in the ISM band. This chip was used due to its low cost, size, and low power consumption as compared to other available options [22]. Each transceiver can use 125 channels with a channel switching time less than 200 ms and data rate of up to 1 Mbps. This implies that 125 different devices can operate in the same environment without interfering with each other.

The assistive device for the blind, given in paper, was first developed for assistance of little children at schools for blind. Therefore, it can have more than 125 users, which can cause problems in communication. Thus, a remedy for limitation in the number of communication channels is required. The number of devices operating in an environment however can be increased by utilizing time division multiple access (TDMA) [23], which however, is not supported by the nRF2401 chip. The device is made to operate in two modes, the first one being the normal mode and the second one crowd mode. The crowd mode utilizes a custom nonstandard TDMA technique. Each device can transmit for 250 ms only whereas the receiver listens throughout and receives data from the transmitter already registered with it. The Probability density function of the uniformly distributed slot interval on an interval with a width (b-a) of 250 ms is given in terms of the Heaviside step function by

(11) $$\begin{array}{c} P\left(s\right)=\frac{H\left(s-a\right)-H\left(s-b\right)}{b-a}. \end{array}$$

The choice of the transmission slot follows a uniform distribution as shown in Equation (11), and in case, a device fails to communicate for 2 seconds in crowd mode, then the randomly generated time slots are shifted to 50 ms repeatedly till successful communication at both ends is achieved. Upon successful communication and built in acknowledgment from the receiver, the message is repeated continuously in the allocated time slot which consists of a start of data identifier (unique for each pair) and data.  Figure 6 depicts a general scenario for crowd mode operation of assistive device. The chip also supports frequency hopping thus enabling the user to implement frequency hopping spread spectrum (FHSS) [23]. Since a pair of Arduinos is used for data processing and communication, frequency hopping is difficult to implement. This is due to the slight difference in the Arduino pair clocks as well as the susceptibility of this low-cost platform to the temperature changes. This practically results in a clock drift and the transceivers getting out of synchronization.

The effectiveness of the assistive device in crowd mode is shown in MATLAB simulation. In Figure 7, the simulation for number of collisions vs. the number of devices is given. It can be seen when the device operates in crowd mode, the number of collisions significantly decreases. The results show how adapting proposed crowd mode technique improved the results several times as compared to the normal mode. Another possible solution to this problem is using a GPS clock for synchronization of the hopping time pattern. This solution can also benefit in the integration of maps with the device and providing the user with a clearer picture of the surroundings. However, due to cost overhead, this idea will be considered for future modifications.

## 4. Experiments and Results

In order to verify the working of device, it is tested while moving on a staircase and under an inclined roof, i.e., under a staircase. Both the belt and ankle module are used, and the scenario is developed such that the user moves on plain surface towards the stair, then he moves on the stairs and at the end he reaches platform. The subject's height for each scenario was 175 cm with the waist sensors installed at a height of 100 cm from the ground and ankle sensors installed at 20 cm from the ground. The average stride length was measured and averaged 32 cm.

In each experiment, the outputs of all sensors are passed through a moving average filter before using them for a decision. The outputs from these sensors after passing through the moving average filter are depicted in Figures 8 and 9. In the first scenario depicted in Figure 8, the subject is climbing stairs. The sensor outputs can be seen to properly register the shape of stairs. The 45°-up sensor is also registering the stairs; however, it is the roof of the staircase which also happened to be inverted stairs. In case of any obstacle classification, the algorithm is designed to gather a data of at least 20 samples and then decide and inform the subject about the upcoming obstacle type when the distance approaches 300 cm or less.  Figure 9 shows the user walking with an incline obstacle upfront. It can be seen that the shape of obstacle has been properly registered by all the ultrasonic sensors and the distance given by each sensor, other than 45°-down sensor, decrease as the user moves.

In order to test performance and effectiveness of the device in real life, statistical experiments are performed. For experimental purpose, a setup is arranged in a 610 × 365 cm^2^ room with static obstacle randomly scattered and three people walking very slowly in it to simulate dynamic obstacles. A person with covered eyes is moved in the room for five minutes. Different sets of experiments, repeated 10 times, are performed; firstly, without any assistive aid; secondly, with a white cane; thirdly, with assistance from only the belt module, and at the end with assistance from both the belt and the ankle modules. The distance, in terms of steps, covered by the person during each experiment along with the number of collisions is calculated separately.

In Figure 10(a), we have given the statistical results of number of collisions in different experiments, plotted in the form of boxplot. It can be seen from the plot that the number of collisions is least when combination of belt and ankle modules is used. On the other hand, by using only the belt module, the number of collisions is slightly more than combined belt-ankle modules. This means that if only the belt module is used, cost can be reduced with expense of slightly more collisions. On the other hand, in Figure 10(b)), we have given the accumulative distance covered, in term of steps taken, during each set of experiment. It can be seen that using both belt and ankle devices resulted in covering of more distance while distance covered without any aid is the least.

In order to analyze the working of device for moving object, we considered case of a vehicle moving in reverse direction and the user of the device standing behind it. The collected data is analyzed in MATLAB. The optimal value for sampling time of *T* = 0.2 s was selected using a hit and trial method. The speed used for the subject is 4.5 km/h [24], whereas the velocity of the object is average reverse speed of a car calculated in campus parking. It was observed that for ultrasonic sensor, with 400 cm range, the response time was about 1 s, which was too small for the state estimator to converge for final range time.

The same experiment was repeated by replacing ultrasonic sensor with a LADAR Lite v3 sensor. The maximum distance used between the moving object and the subject was chosen corresponding to the maximum range of the LADAR Lite v3 sensor which is 40 m with a three-sigma bound of 3 cm in each direction. The trajectories of the vehicle in reverse and a subject with the proposed device are depicted in Figure 11. In Figure 12, we have given the root mean square error (RMSE) of the range, range rate, and the time to react using a Kalman filter. Since the time to react becomes shorter, the warning beep interval is reduced to warn the subject about an imminent collision with the moving object. However, it is better than that of ultrasonic sensor.

## 5. Conclusion Remarks

In this paper, we have given the design and construction of a new assistive device for visually impaired people. It is of low cost and uses ultrasonic sensors and IMU to obtain information about surroundings. Unlike other such devices that uses ultrasonic sensors, this device has more features where it can distinguish position of obstacles as well as can detect different types of obstacles at different positions in front of the user. The device can detect obstacle at head level, in front, and at ground. At the end, experiments are done to check the statistical advantages of the new device. It was seen that the newly constructed assistive device performs better as compared to conventional assistive methods. The modular form of the device has increased the choice for the user. The user can only purchase one module at lesser price and lose only few features. The other module can also be added in the same first module after some time. The use of voice instruction was a new method of communication with the user, in which clear instructions can be added by the user in his/her own voice.

In order to get better response time for fast moving objects, the front ultrasonic sensor was replaced by LADAR Lite v3 sensor. It was observed that the LADAR gave better results. However, this has increased the cost of the device. The comparison of existing range sensor-based assistive devices for visually impaired people with our device is given in Table 1. It can be observed that our device provides better features than other devices. In the near future, camera for vision-based assistance will be added in the proposed device.

## Figures and Tables

**Figure 1:** Different mobility assistive devices for visually impaired people: (a) [18], (b) [11], (c) [15], and (d) [7].

**Figure 2:** Evaluation for design consideration of an assistive device for visually impaired people. (a) Layout of the device. (b) Obstacle at head level. (c) A pit hole on a straight path. (d) Obstacle upfront. (e) Stairs or small obstacle in front.

**Figure 3:** Architecture for modular assistive device for visually impaired people.

**Figure 4:** Newly constructed modular assistive device: (a) belt module and (b) ankle module.

**Figure 5:** The moving average filter used as a low-pass filter for the raw sensor input.

**Figure 6:** The customized protocol for multiple users in crowd mode.

**Figure 7:** Number of devices vs. number of collisions.

**Figure 8:** Actual sensor measurements after passing through a moving average filter (stairs).

**Figure 9:** Actual sensor measurements after passing through a moving average filter (inclined obstacle up ahead).

**Figure 10:** Statistical results: (a) number of cotillions and (b) distance covered. (1) Without any aid, (2) with cane, (3) with belt module only, and (4) with belt and ankle module.

**Figure 11:** Collision trajectory of the moving object and subject with proposed device.

**Figure 12:** Root mean square errors from the estimation process for trajectories depicted in Figure 11. (a) Range and range rate. (b) Time to react.

**Algorithm 1:** Algorithm for working of the proposed assistive device.

**Table 1:** Comparison of range-based assistive device with the device presented in the paper.

Author	[14]	[15]	[16]	[17]	[25]	[26]	Our device
Range	Small	Medium	Medium	Medium	Medium	Large	Medium
Cost	High	Low	High	High	Low	High	Low
Weight	Heavy	Light	Heavy	Heavy	Light	Heavy	Light
Obstacle detection	Front	Front	Front	Front	Front	Front	Front-up-down
Stair detection	Yes	No	No	No	No	No	Yes
Instructions	No	No	No	No	No	No	Yes

## Data Availability

The data can be provided on demand.
